The article "Therapeutic effects of bone marrow-derived mononuclear cells from healthy or silicotic donors on recipient silicosis mice" was published in 2017. Journal: Stem Cell Res Ther.

# Therapeutic effects of bone marrow-derived mononuclear cells from healthy or silicotic donors on recipient silicosis mice

**DOI:** 10.1186/s13287-017-0699-7

**Published:** 2017-11-10

**Authors:** Helena D’Anunciação de Oliveira, Elga Bernardo Bandeira de Melo, Johnatas Dutra Silva, Jamil Zola Kitoko, Bianca Gutfilen, Thiago Barboza, Sergio Augusto Lopes de Souza, Christina Maeda Takiya, Patricia Rieken Macedo Rocco, Miquéias Lopes-Pacheco, Marcelo Marcos Morales

**Affiliations:** 1 Laboratory of Cellular and Molecular Physiology, Carlos Chagas Filho Institute of Biophysics, Federal University of Rio de Janeiro, Rio de Janeiro, Brazil; 2 Laboratory of Pulmonary Investigation, Carlos Chagas Filho Institute of Biophysics, Federal University of Rio de Janeiro, Rio de Janeiro, Brazil; 3 Department of Radiology, School of Medicine, Federal University of Rio de Janeiro, Rio de Janeiro, Brazil; 4 Laboratory of Cellular Pathology, Carlos Chagas Filho Institute of Biophysics, Federal University of Rio de Janeiro, Rio de Janeiro, Brazil

**Keywords:** Silicosis, Cell therapy, Bone marrow mononuclear cells, Lung fibrosis, Inflammation

## Abstract

**Background:**

Administration of bone marrow mononuclear cells (BMMCs) modulates lung inflammation and fibrosis in experimental silicosis. However, no studies have evaluated whether silicosis affects the efficacy of autologous BMMCs treatment. We hypothesized that BMMCs obtained from healthy or silicotic mice may improve lung function, but they might affect the inflammatory and fibrotic processes differently in experimental silicosis.

**Methods:**

C57BL/6 mice were randomly divided into control (C) and silicosis (SIL) groups. Mice in the SIL group were instilled with silica particles intratracheally; the C animals received saline using the same protocol. On day 15, the animals were treated with saline (Sal) or BMMCs (2 × 10^6^ cells) from healthy (BMMC-healthy) and silicotic (BMMC-sil) donors. Lung mechanics were measured, and lungs were collected for histology and molecular biology analysis.

**Results:**

BMMCs obtained from healthy and silicotic donors presented similar percentages of cell populations. ^99m^Tc-BMMCs tracking revealed preferential migration of cells to the liver, and only a few GFP^+^ BMMCs were observed in lung tissue 24 h after treatment, regardless of donor type. Both the SIL-BMMC-healthy and SIL-BMMC-sil groups showed improvement in lung function, a reduction in the fractional area of granuloma, and a decrease in the number of mononuclear and apoptotic cells in lung parenchyma. In addition, the number of F4/80^+^ macrophages, the levels of interleukin-1 beta and transforming growth factor beta, and collagen fiber content in granuloma were reduced in SIL-BMMC-healthy mice, whereas mRNA expression of MMP-9 and procollagen I and III was reduced in the SIL-BMMC-sil group.

The article "Therapeutic effects of bone marrow-derived mononuclear cells from healthy or silicotic donors on recipient silicosis mice" was published in 2017. Journal: Stem Cell Res Ther.

**Conclusions:**

Administration of BMMCs from healthy and silicotic donors reduced lung inflammation and fibrosis, thus improving lung function. In addition, BMMC-healthy exhibited a greater improvement in lung morpho-functional changes in murine model of silicosis.

## Background

Crystalline silica particles are highly polymorphic molecules, commonly found as quartz or sand. Inhalation of these particles triggers an inflammatory process and culminates in lung fibrosis [1–3]. Silica particles impair lung clearance and their continuous stimuli result in persistent inflammation [4, 5], which is characterized by leukocyte infiltration and release of chemokines, pro-inflammatory cytokines, and proteolytic enzymes that cause disruption of the extracellular matrix (ECM) [6]. In this context, upregulation of matrix metalloproteinase (MMP) expression, massive production of collagen, and release of cytokines related to the fibrotic response, such as interleukin (IL)-1β and tumor necrosis factor (TNF)-α, result in interstitial fibrosis [7]. Although mortality has decreased globally in the last decades, silicosis is still prevalent in developing countries, especially in China, South Africa, and Brazil [3], where approximately 6 million workers are continuously exposed to silica particles [8, 9]. To date, there is no curative treatment for silicosis, and new therapies have been sought to improve the quality of life and life expectancy of patients with silicosis [3].

In previous studies conducted by our group, we have observed that prophylactic administration of bone marrow mononuclear cells (BMMCs) reduced mRNA expression of pro-inflammatory and pro-fibrotic mediators [10]. In addition, therapeutic administration of BMMCs mitigated lung fibrosis in the late stage of silicosis [11]. BMMCs therapy has some advantages compared with other cell-based treatments: (1) it does not require cell-culture processes, which reduces the costs related to the treatment; (2) it does not have a risk of cellular rejection; and (3) it could be used in autologous transplantation. However, the effects of the continuous inflammatory stimuli observed during silicosis on the profile of BMMC populations remain unclear, as well as the effects of these cells as a therapeutic approach.

To answer this open question, we have evaluated the therapeutic effects of BMMCs obtained from healthy and silicotic donors on lung mechanics, inflammation, and remodeling in murine model of silicosis. We hypothesized that BMMCs from healthy donors may have greater effects on lung inflammation and fibrosis than BMMCs from silicotic donors, although both could improve lung mechanics. For this purpose, BMMCs obtained from healthy and silicotic mice were characterized and then intravenously administered to silicotic animals.

The article "Therapeutic effects of bone marrow-derived mononuclear cells from healthy or silicotic donors on recipient silicosis mice" was published in 2017. Journal: Stem Cell Res Ther.

## Methods

### Experimental protocol

A total of 135 male and female C57BL/6 mice (20–25 g, 8–12 weeks old) were used. Female mice received 50 μL of 0.9% sterile saline intratracheally (control group [C]) or 20 mg of silica (Sigma-Aldrich, St. Louis, MO, USA) in 50 μL of saline (silicosis group [SIL]). Fifteen days after saline or silica instillation, the C and SIL groups were further randomized into subgroups receiving an intravenous injection of 50 μL of saline (Sal) or BMMCs (2 × 10^6^ cells/50 μL of saline) obtained from healthy (BMMC-healthy) or silicotic (BMMC-sil) male donors in the internal jugular vein.

### Extraction of BMMCs

C57BL/6 male mice received saline or silica as described above. On day 15, bone marrow was harvested from the femur and tibia with Dulbecco’s modified Eagle’s medium (DMEM; Life Technologies, Camarillo, CA, USA). After a homogeneous cell suspension was achieved, cells were centrifuged (400 × *g* for 10 min), re-suspended in DMEM, and added to Ficoll-Hypaque gradient (Histopaque 1083; Sigma Chemical Co., St. Louis, MO, USA). The cells isolated from the gradient interface corresponding to putative mononuclear cells were counted in a Neubauer chamber with trypan blue for evaluation of viability. The same protocol was applied for extraction of BMMCs derived from green fluorescent protein (GFP)^+^ mice.

### Flow cytometry

BMMCs derived from healthy or silicotic (sil) animals were pooled to achieve samples of ten million cells. Thereafter, BMMCs were isolated by Ficoll-Hypaque density gradient centrifugation, and subpopulations were characterized by flow cytometry using specific surface antibodies to detect: mesenchymal stem cells (MSCs) (CD44^+^/CD29^+^/CD45^−^/CD11b^−^), hematopoietic stem cells (HSCs) (CD34^+^/CD45^−^/CD11b^−^) monocytes (CD45^+^/CD11b^+^), neutrophils (SSC^high^/GR^+^/Siglec^−^), T lymphocytes (CD45^+^/CD3^+^/B220^−^), T helper (Th) lymphocytes (CD45^+^/CD3^+^/CD4^+^/B220^−^), and B lymphocytes (CD45^+^/B220^+^). All antibodies were purchased from BD Biosciences (San Diego, CA, USA) and used according to the manufacturer’s instructions. Data were acquired on a BD FACSCalibur cytometer (Becton Dickinson, Mansfield, MA, USA) and analyzed by Cellquest and PAINT-A-GATE software.

### Biodistribution of BMMCs labeled with ^99m^Technetium (^99m^Tc)

BMMCs were labeled with ^99m^Tc following protocols described previously by our group [12, 13]. Briefly, 500 μL of sterile SnCl_2_ solution was added to a cell suspension, and the mixture was incubated at room temperature for 10 min. Then, 5 mCi of ^99m^Tc was added, and the incubation was continued for another 10 min. After centrifugation (500 × *g* for 5 min), the supernatant was removed, and the cells were washed three times with 0.9% saline. Viability of the labeled cells was assessed by trypan blue and was estimated to be greater than 93% in all cases. Labeling efficiency (%) was calculated by the activity in the pellet divided by the sum of the radioactivity in the pellet plus the supernatant, and was estimated to be greater than 90% in all cases. 2 × 10^6^ ^99m^Tc-BMMCs were intravenously injected by jugular vein immediately after labeling. For analysis of qualitative biodistribution, whole-body scintigraphy was performed on the animals through a dedicated small-animal microSPECT/CT camera (Triumph, Trifoil, Los Angeles, CA, USA) equipped with a high-resolution collimator and diagnostic computed tomography (CT) 2 h after ^99m^Tc-BMMC administration.

The article "Therapeutic effects of bone marrow-derived mononuclear cells from healthy or silicotic donors on recipient silicosis mice" was published in 2017. Journal: Stem Cell Res Ther.

### Lung mechanics

Thirty days after saline or silica instillation, animals were sedated (diazepam, 1 mg intraperitoneally [i.p.]), anesthetized (thiopental sodium, 20 mg/kg, i.p.), tracheotomized, paralyzed (vecuronium bromide, 0.005 mg/kg, intravenously [i.v.]), and mechanically ventilated with a constant flow ventilator (Samay VR15; Universidad de la Republica, Montevideo, Uruguay) using the following parameters: tidal volume, 0.2 mL; respiratory rate, 100 breaths/min; and fraction of inspired oxygen, 0.21. The anterior chest wall was surgically removed and a positive end-expiratory pressure of 2 cm H_2_O was applied. In an open-chest preparation, tracheal pressure reflects transpulmonary pressure. Static lung elastance (Est,L), the pressure spent to overcome airway resistance (ΔP1,L), and stress relaxation or viscoelastic properties of the lung (ΔP2,L) were measured using ANADAT data analysis software (RHT-InfoData, Inc., Montreal, QC, Canada).

### Lung histology

Immediately after the determination of lung mechanics, laparotomy was performed and heparin (1,000 IU i.v.) was injected. The trachea was clamped at end expiration, and the abdominal aorta and vena cava were sectioned. The left lung was then isolated, quickly frozen by immersion in liquid nitrogen, fixed with Carnoy’s solution, and embedded in paraffin. Slices were cut (4 μm thick), deparaffinized, and stained with hematoxylin and eosin. The fractional area of granuloma and the total and differential cellularity in the lung tissue were determined by the point-counting technique at a magnification of ×200 and ×1000, respectively, across ten random, non-coincident microscopic fields [14].

The article "Therapeutic effects of bone marrow-derived mononuclear cells from healthy or silicotic donors on recipient silicosis mice" was published in 2017. Journal: Stem Cell Res Ther.

Diffuse alveolar damage was quantified using a weighted scoring system by a researcher blinded to the experimental protocol [15]. Briefly, scores of 0 to 4 were used to represent septal thickening with 0 standing for no effect and 4 for maximum severity. In addition, the extent of each scored characteristic per field of view was determined on a scale of 0 to 4, with 0 standing for no visible evidence and 4 for complete involvement. Scores were calculated as the product of severity and the extent of each feature, and thus ranged from 0 to 16. Scoring was assessed by one pathologist expert in lung histology. The assessor was blinded to group assignment.

Collagen fibers were quantified using Sirius red staining. Ten microscopic fields in lung parenchyma and granulomas were randomly selected, and high-quality images were captured at a magnification of ×400, after setting and calibrating the Q Capture pro 4.5 software (QImaging, Surrey, BC, Canada). The content of collagen fibers was measured using Image Pro Plus 4.5.1 software (Media Cybernetics, Rockville, MD, USA).

Immunohistochemistry was performed in paraffin sections to quantify macrophages and GFP^+^ cells using the following antibodies: monoclonal antibody F4/80 rat anti-mouse (cat. no. MCA497; AbDSerotec, Raleigh, NC, USA) and GFP rabbit IgG polyclonal antibody fraction (cat. no. A-11122; Life Technologies). Secondary antibody labeled with peroxidase from Histofine simple stain for mouse tissue, anti-rat (immuno-enzyme polymer with peroxidase; Nichirei Biosciences Inc., Tokyo, Japan) followed by chromogen substrate diaminobenzidine (DAB liquid, cat. no. K3468; Dakocytomation, Carpinteria, CA, USA) were used to detect the specific antibodies described above. Quantification was performed in 20 random and non-coincident microscopic fields (magnification of ×400). Images were analyzed by manual cell counting using the multi-point tool in ImageJ software [16]. The results are expressed as the percentage of positive cells per total cells in microscopic fields.

### In situ apoptosis

Apoptotic cells in lung tissue were detected by terminal deoxynucleotidyl transferase biotin-dUTP nick end labeling (TUNEL) assay, according to the manufacturer’s instructions (cat. no. S7100; EMD Millipore, Billerica, MA, USA). Twenty fields from alveolar septa and granuloma were randomly selected, images were acquired (magnification of ×400) and then analyzed using ImageJ software, as described above. The results are expressed as the percentage of positive cells per total cells in the microscopic fields.

### Enzyme-linked immunosorbent assay

Levels of IL-1β, TNF-α, IL-6 (Peprotech, Rocky Hill, NJ, USA), transforming growth factor (TGF)-β (R&D Systems, Minneapolis, MN, USA), and IL-10 (BD Biosciences, San Diego, CA, USA) were quantified in homogenate lung tissue by ELISA according to the manufacturer’s instructions.

The article "Therapeutic effects of bone marrow-derived mononuclear cells from healthy or silicotic donors on recipient silicosis mice" was published in 2017. Journal: Stem Cell Res Ther.

### Real-time reverse transcription-polymerase chain reaction

Quantitative real-time RT-PCR was performed to measure the relative expression levels of mediators associated with lung remodeling. Total RNA was extracted from the frozen tissues using an RNeasy Mini Kit (cat. no. 74106; Qiagen, Hilden, Germany) according to the manufacturer’s recommendations. The RNA concentration was measured by spectrophotometry in Nanodrop 2000c (Thermo Fisher Scientific, Wilmington, DE, USA). First-strand cDNA was synthesized from total RNA using a QuantiTect Reverse Transcription Kit (cat. no. 205314; Qiagen). PCR primers for the target gene were purchased from Invitrogen (Carlsbad, CA, USA). Expression of the target genes was normalized to a control gene (acidic ribosomal phosphoprotein P0 [36B4]), and the relative fold changes were calculated using the ΔΔC_T_ method. The following PCR primers were used: type I procollagen, forward: 5′-TGA CTG GAA GAG CGG AGA GT-3′, reverse: 5′-GTT CGG GCT GAT GTA CCA GT-3′; type III procollagen, forward: 5′-GTG GGA CCT GGT TTC TCA CCC T-3′, reverse: 5′-GGT TGG GGC AGT CTA GTG GCT C-3′; metalloprotease (MMP)-9, forward: 5′-AGT CCG GCA GAC AAT CCT T-3′, reverse: 5′- CCC TGT AAT GGG CTT CCT C-3′; 36B4, forward: 5′-CAA CCC AGC TCT GGA GAA AC-3′, reverse: 5′-GTT CTG AGC TGG CAC AGT GA-3′.

### Statistical analysis

The normality of the data was tested using the Kolmogorov-Smirnov test with Lilliefors correction. The Levene median test was used to evaluate the homogeneity of variances. If both conditions were satisfied, one-way ANOVA followed by Tukey’s post hoc test or two-way ANOVA followed by Bonferroni’s test was used. The Kruskal-Wallis test followed by Dunn’s test was used to compare non-parametric data. Parametric data are expressed as means ± standard deviation (SD), and non-parametric data are expressed as medians (interquartile range). Student’s *t* test was used to compare the flow cytometry data. All tests were performed using the Prism 6.7 software package (GraphPad Software Inc., La Jolla, CA, USA). In all tests, the significance level was set at 5%.

## Results

### Characterization and biodistribution of BMMCs

BMMCs derived from healthy or silicotic donors were characterized by flow cytometry. No significant differences in HSCs and MSCs populations, as well as in monocytes, B lymphocytes, T lymphocytes, and eosinophils, were observed in BMMCs obtained from both type of donors (Fig. 1).

The article "Therapeutic effects of bone marrow-derived mononuclear cells from healthy or silicotic donors on recipient silicosis mice" was published in 2017. Journal: Stem Cell Res Ther.

**Fig. 1:** Flow cytometry of bone marrow mononuclear cells. Absolute values of total cells (**a**), monocytes (**b**), neutrophils (**c**), mesenchymal stem cells (*MSCs*) (**d**), hematopoietic stem cells (*HSCs*) (**e**), B lymphocytes (**f**), T lymphocytes (**g**), CD4^+^ T lymphocytes (**h**), eosinophils (**i**) in the BMMC population. n = 6 per group

Biodistribution was analyzed using BMMCs from healthy and silicotic (sil) donors labeled with ^99m^Tc and then injected into the jugular vein of control (C) or silicotic (SIL) recipients. Images obtained 2 h after injection showed cell migration preferentially to the liver (Fig. 2a). In addition, only a few GFP^+^ BMMCs were observed in lung tissue 24 h after intravenous injection in animals in both the SIL-BMMC-healthy and SIL-BMMC-sil groups (Fig. 2b).

**Fig. 2:** Biodistribution and homing of bone marrow mononuclear cells (*BMMCs*). **a** Representative coronal whole-body SPECT/CT images of control (*C*) and silicotic (*SIL*) animals 2 h after intravenous administration of ^99m^Tc-BMMCs derived from heathy or silicotic (*sil*) donors. ^99m^Tc-BMMCs migrate to the liver in all experimental groups (Li). *B* bladder. n = 4 animals per group. **b** Representative photomicrographs of lung parenchyma, granuloma, and spleen after immunohistochemistry with green fluorescent protein (*GFP*) antibody. Rare inflammatory GFP^+^ cells (*black arrows*) were observed in lung parenchyma and in granulomas of the SIL-BMMC groups 24 h after treatment with BMMCs from GFP^+^ mice. Spleens of GFP male mice were used as positive control. Bars, 100 μm. n = 4 animals per group

### BMMCs derived from healthy and silicotic donors improved lung function in experimental silicosis

Est,L, ΔP1,L, and ΔP2,L were similar in the C-Sal, C-BMMC-healthy, and C-BMMC-sil groups (Fig. 3). SIL-Sal mice presented increased Est,L, ΔP1,L, and ΔP2,L compared with mice in the C groups. Both SIL-BMMC-healthy and SIL-BMMC-sil animals showed decreased Est,L and ΔP2 compared with SIL-Sal animals, with ΔP2 presenting similar levels to that observed in the C-Sal group. The SIL-BMMC-healthy group, but not the SIL-BMMC-sil group, presented a reduction in ΔP1 compared with SIL-Sal.

**Fig. 3:** Lung mechanics. Lung static elastance (Est,L) (**a**), resistive (ΔP1,L) and viscoelastic (ΔP2,L) pressures (**b**). Control (*C*) and silicotic (*SIL*) mice received saline (*Sal*)(50 μL) or silica (20 mg silica/50 μL saline) intratracheally. C and SIL animals were treated with bone marrow mononuclear cells (BMMCs) derived from healthy or silicotic (*sil*) donors. Values are means ± SD. n = 10 animals in each group. ^*^Significantly different from C-Sal (*P* < 0.05). ^#^Significantly different from Sil-Sal (*P* < 0.05)

The article "Therapeutic effects of bone marrow-derived mononuclear cells from healthy or silicotic donors on recipient silicosis mice" was published in 2017. Journal: Stem Cell Res Ther.

### BMMCs derived from healthy and silicotic donors mitigated lung inflammation and remodeling differently in experimental silicosis

C groups showed preserved lung structure, whereas intratracheal instillation of crystalline silica led to morphological alterations in lung parenchyma, characterized by an increased number of inflammatory cells and alveolar wall thickening, as well as the presence of granuloma (Table 1, Fig. 4). SIL-BMMC-healthy and SIL-BMMC-sil mice, compared with SIL-Sal mice, presented a reduction in the total and mononuclear cell counts. Only animals in the SIL-BMMC-healthy group showed a reduced polymorphonuclear cell count in lung parenchyma. In addition, both SIL-BMMC-healthy and SIL-BMMC-sil groups presented a reduction in the total and polymorphonuclear cell counts, as well as the fractional area of granuloma. Only the mice in the SIL-BMMC-sil group showed a decreased number of mononuclear cells in granulomas. Neither BMMC-healthy nor BMMC-sil reduced alveolar wall thickening. Because we did not observe differences in lung function and histology among the C-Sal, C-BMMC-healthy, and C-BMMC-sil groups, we used only C-Sal mice to perform the following experiments.

**Table 1:** Lung inflammation: total number of cells, number of mononuclear and polymorphonuclear cells in lung tissue

	MN (%)	PMN (%)	Total (%)
Lung parenchyma			
C-Sal	35.8 ± 3.3	5.8 ± 1.6	41.6 ± 3.1
C-BMMC-healthy	37.0 ± 4.3	5.2 ± 2.3	42.2 ± 5.1
C-BMMC-sil	33.1 ± 3.1	6.0 ± 1.9	39.1 ± 3.8
SIL-Sal	42.6 ± 3.3^*^	8.2 ± 2.3	50.9 ± 2.9^*^
SIL- BMMC-healthy	38.3 ± 4.4^#^	5.1 ± 2.8^#^	43.3 ± 4.2^#^
SIL- BMMC-sil	35.3 ± 2.1^#^	5.8 ± 3.3	41.2 ± 4.2^#^
Granuloma			
SIL-Sal	38.8 ± 1.5	11.3 ± 2.3	50.1 ± 2.0
SIL- BMMC-healthy	36.2 ± 2.8	7.2 ± 3.2^#^	43.5 ± 4.3^#^
SIL- BMMC-sil	34.2 ± 2.5^#^	6.8 ± 2.7^#^	41.0 ± 3.7^#^

Control (C) and silicotic (SIL) mice received saline (50 μL) or silica (20 mg silica/50 μL saline) (Sal) intratracheally. C and SIL animals were treated with bone marrow mononuclear cells (BMMCs) (2 × 10^6^ cells) derived from healthy or silicotic (sil) donors. *MN* mononuclear cells, *PMN* polymorphonuclear cells, *total* total cellularity. Values are means ± SD. N = 10 animals per group. ^*^Significantly different from C-Sal (*P* < 0.05). ^#^Significantly different from SIL-Sal (*P* < 0.05)

**Fig. 4:** Representative photomicrographs of lung parenchyma stained with hematoxylin and eosin (**a**) of C-Sal, SIL-Sal, SIL-BMMC-healthy, and SIL-BMMC-sil groups. (**b**) Quantification of the fractional area of granuloma. (**c**) Diffuse alveolar damage analysis. Control (*C*) and silicotic (*SIL*) mice received saline (*Sal*) or silica and were then treated with bone marrow mononuclear cells (BMMCs) obtained from healthy or silicotic (*sil*) donors. Note the presence of granulomas (^*^) in the SIL groups. Values are means ± SD. n = 9 animals in each group. Bars, 100 μm. ^*^Significantly different from C-Sal (*P* < 0.05). ^#^Significantly different from SIL-Sal (*P* < 0.05)

Macrophages have a crucial role in the pathophysiology of silicosis. Alveolar macrophages are stimulated by silica particles to release mediators involved in the recruitment of inflammatory cells and activation of fibroblasts [17]. Animals in the SIL-Sal group presented an increased number of F4/80^+^ macrophages in lung parenchyma compared with the C-Sal group (Fig. 5). SIL-BMMC-healthy mice, but not SIL-BMMC-sil mice, exhibited a lower number of F4/80^+^ macrophages in lung granulomas compared with SIL-Sal mice. Associated with the increased number of F4/80^+^ macrophages, IL-1β levels were increased in SIL-Sal mice compared with C-Sal mice (Fig. 6a). SIL-BMMC-healthy mice, but not SIL-BMMC-sil mice, presented decreased levels of IL-1β compared with SIL-Sal mice. BMMC-healthy or BMMC-sil therapy was not able to reduce IL-6 and TNF-α protein levels in SIL mice (data not shown). SIL-BMMC-healthy mice presented similar IL-10 protein levels compared with SIL-Sal mice, whereas it was reduced in SIL-BMMC-sil group (Fig. 6b).

The article "Therapeutic effects of bone marrow-derived mononuclear cells from healthy or silicotic donors on recipient silicosis mice" was published in 2017. Journal: Stem Cell Res Ther.

**Fig. 5:** Representative photomicrographs of lung parenchyma after immunohistochemistry with F4/80 (**a**) antibody. F4/80^+^ macrophages were quantified in lung parenchyma (**b**) and granuloma (**c**), and represented as percentage of positive cells. n = 6 animals in each group. Bars, 100 μm. ^*^Significantly different from C-Sal (*P* < 0.05). ^#^Significantly different from Sil-Sal (*P* < 0.05). *BMMC* bone marrow mononuclear cell, *C* control, *Sal* saline, *SIL* silicotic mice, *sil* treated with BMMCs derived from silicotic donors

**Fig. 6:** Protein levels of IL-1β, IL-10 and TGF-β in lung tissue. Protein levels of (**a**) interleukin (*IL*)-1β, (**b**) IL-10 and (**c**) transforming growth factor (*TGF*)-β were quantified in lung tissue. Values are means ± SD. n = 5–8 animals per group. ^*^Significantly different from C-Sal (*P* < 0.05). ^#^Significantly different from Sil-Sal (*P* < 0.05). ^&^Significantly different from SIL-BMMC-healthy (*P* < 0.05). *BMMC* bone marrow mononuclear cell, *C* control, *Sal* saline, *SIL* silicotic mice, *sil* treated with BMMCs derived from silicotic donors

Increased secretion of growth factors, such as TGF-β, leads to fibroblast proliferation and collagen deposition to replace the damaged tissue. In addition, silica-induced lung fibrosis is associated with dysregulated expression of MMPs and their inhibitors [18]. Protein levels of TGF-β, as well as mRNA levels of procollagen III and I, and MMP-9, were increased in the SIL-Sal group compared with the C-Sal group (Figs. 6c and 7). SIL-BMMC-healthy mice presented reduced protein levels of TGF-β, whereas SIL-BMMC-sil mice showed decreased mRNA levels of procollagen III and I, and MMP-9.

The article "Therapeutic effects of bone marrow-derived mononuclear cells from healthy or silicotic donors on recipient silicosis mice" was published in 2017. Journal: Stem Cell Res Ther.

**Fig. 7:** mRNA levels of type III and I procollagens, MMP-9 in lung tissue. Real-time RT-PCR analysis of mRNA of (**a**) type III and (**b**) type I procollagen, and (**c**) matrix metalloproteinase (*MMP*)-9. Values are means ± SD. n = 8 animals in each group. ^*^Significantly different from C-Sal (*P* < 0.05). ^#^Significantly different from Sil-Sal (*P* < 0.05). *BMMC* bone marrow mononuclear cells, *C* control, *Sal* saline, *SIL* silicotic mice, *sil* treated with BMMCs derived from silicotic donors

Collagen content was increased in SIL-Sal mice compared with C-Sal mice (Fig. 8). SIL-BMMC-healthy group, but not SIL-BMMC-sil group, presented reduced collagen content in granulomas compared with the SIL-Sal group.

**Fig. 8:** Representative photomicrographs of lung parenchyma stained with Sirius red (**a**) from animals in the C-Sal, SIL-Sal, SIL-BMMC-healthy, and SIL-BMMC-sil groups. Collagen fibers were quantified in (**b**) lung parenchyma and (**c**) granuloma. Values are means ± SD. n = 6 animals per group. Bars, 100 μm. ^*^Significantly different from C-Sal (*P* < 0.05). ^#^Significantly different from SIL-Sal (*P* < 0.05). *BMMCs* bone marrow mononuclear cells, *C* control, *Sal* saline, *SIL* silicotic mice, *sil* treated with BMMCs derived from silicotic donors

### BMMCs derived from healthy and silicotic donors mitigated apoptosis of lung parenchyma cells

Silica instillation led to a significant increase in apoptotic cell count in lung tissue compared with the C-Sal group (Fig. 9). Both SIL-BMMC-healthy and SIL-BMMC-sil groups, compared with the SIL-Sal group, showed a reduction in the number of apoptotic cells in the lung parenchyma, but not in granulomas.

**Fig. 9:** Representative photomicrographs of lung parenchyma stained after TUNEL assay (**a**) in the C-Sal, SIL-Sal, SIL-BMMC-healthy, and SIL-BMMC-sil groups. Apoptotic cells (*arrows*) were quantified in (**b**) lung parenchyma and (**c**) granuloma. n = 4 animals in each group. Scale bars, 100 μm. ^*^Significantly different from C-Sal (*P* < 0.05). ^#^Significantly different from SIL-Sal (*P* < 0.05). *BMMCs* bone marrow mononuclear cells, *C* control, *Sal* saline, *SIL* silicotic mice, *sil* treated with BMMCs derived from silicotic donors

The article "Therapeutic effects of bone marrow-derived mononuclear cells from healthy or silicotic donors on recipient silicosis mice" was published in 2017. Journal: Stem Cell Res Ther.

## Discussion

In the present study, we have evaluated the therapeutic effects of BMMCs obtained from healthy and silicotic mice on lung function, as well as inflammatory and remodeling processes in experimental silicosis. Silicosis is marked by persistent inflammation, which results in tissue damage and remodeling. The pathophysiology process is characterized by an influx of leukocytes into lung parenchyma, release of inflammatory mediators, activation and proliferation of fibroblasts, and imbalance between the synthesis and degradation of ECM. Progressive lung fibrosis causes impairment of lung function, leading to death as a result of respiratory failure. To date, there is no treatment to halt or reverse the progression of the disease and reduce the mortality rate. Therefore, new therapies have been sought to mitigate the morpho-functional changes and improve life expectancy and quality of life of patients with silicosis [1, 3, 19].

Cell-based therapy has been studied in different models of lung disease. It has been demonstrated that MSCs administration decreased expression levels of pro-inflammatory and pro-fibrotic mediators as well as tissue remodeling in a model of bleomycin-induced lung injury [20, 21]. In addition, other studies have shown that cell-based therapy modulated lung inflammation and fibrosis in an experimental model of silicosis and lung fibrosis [10, 11, 21–24]. In this context, BMMCs administration represents an interesting alternative, because it does not require cell-culturing processes and there is no risk of transplant rejection. In previous studies from our group, we have shown that BMMCs administration, in a prophylactic or therapeutic manner, improved lung function by reducing lung inflammation [10] and fibrosis [11]. However, no study was performed to comparatively evaluate the therapeutic potential of BMMCs derived from both silicotic and healthy donors in experimental silicosis.

BMMCs characterization performed by flow cytometry revealed no differences between cells pooled from silicotic or healthy donors. A classic study using bone marrow specimens obtained from silicotic volunteers revealed that monocytes and lymphocytes remain within the normal range [25], which corroborates our findings. The same report has described a subtle increase in eosinophils, as well as a marked hyperplasia in bone marrow, in contrast to our findings. Although our model of silicosis mimics the lung damage observed in humans, these conflicting results may be attributed to the time of silica exposure and its continuous stimuli for years in humans, whereas our analysis was performed only 15 days after silica instillation in mice. In addition, we observed similarity in the absolute numbers of MSCs and HSCs in the bone marrow mononuclear population from silicotic and healthy animals.

The article "Therapeutic effects of bone marrow-derived mononuclear cells from healthy or silicotic donors on recipient silicosis mice" was published in 2017. Journal: Stem Cell Res Ther.

Analysis of the biodistribution was carried out using ^99m^Tc, which efficiently labels the mononuclear fraction of bone marrow cells and allows cell tracking after systemic injection [26]. Two hours after administration, both ^99m^Tc-BMMC-healthy and ^99m^Tc-BMMC-sil migrated preferentially to the liver in the SIL and C groups. Because of the relative short half-life of ^99m^Tc of 6 h [26], immunohistochemistry for GFP^+^ BMMCs was performed 24 h after treatment. We observed only a few GFP^+^ BMMCs in lung tissue in both the SIL-BMMC-healthy and SIL-BMMC-sil groups. These data suggest that BMMCs derived from silicotic or healthy donors act systemically, and cell engraftment in lung tissue is not required to obtain therapeutic effects in silicosis.

Impairment of lung mechanics is observed after intratracheal instillation of silica, and it may be correlated to infiltration of inflammatory cells and collagen deposition in lung tissue [4]. In this context, similar improvements in Est,L and ΔP2 were observed after administration of both BMMC-healthy or BMMC-sil in SIL mice. This may be associated with the reduction in polymorphonuclear cell counts and the fractional area of granuloma. Importantly, only SIL-BMMC-healthy was able to improve ΔP1, which may be correlated with a reduction in the inflammatory and remodeling processes in the airways.

The increasing number of mononuclear cells observed after silica instillation led us to further investigate the recruitment of macrophages in lung tissue. Macrophages play a crucial role in the pathophysiology of silicosis by secreting pro-inflammatory mediators, such as IL-1β, TNF-α, IL-6, MIP-1, and MIP-2, as well as growth factors and fibrogenic mediators, which lead to fibroblast activation and collagen deposition [27]. Among these mediators, IL-1β is a pivotal inflammatory cytokine produced by macrophages [28]. In this context, the decreased IL-1β levels in lung tissue in the SIL-BMMC-healthy group may be correlated with a reduced F4/80^+^ macrophage count in this same group. On the other hand, SIL-BMMC-sil mice did not present a reduction in IL-1β levels or in the recruitment of macrophages in lung tissue. Thus, the reduction of mononuclear cell counts after BMMC-sil treatment could be related to changes in lymphocyte populations.

An increase in IL-1β levels might stimulate epithelial-mesenchymal transition and myofibroblast activation through a TGF-β1-mediated mechanism, thus leading to lung fibrosis [29]. The fibrotic process involves modified expression of matrix-degrading-related enzymes, as well as secretion of TGF-β and platelet-derived growth factor [30]. In the present study, the SIL-BMMC-healthy group showed a reduction in TGF-β levels in lung tissue compared with SIL-Sal mice. Min et al. [31] observed that human umbilical cord-derived MSCs decreased TGF-β, MMP-9, and collagen I expression, as well as tissue remodeling in a murine model of bleomycin-induced lung fibrosis. Furthermore, our group has previously shown that prophylactic administration of BMMCs reduced mRNA levels of TGF-β, IL-1β, IL-1α, and IL-1RN and attenuated silica-induced lung fibrosis [10]. However, in a chronic model of silicosis, BMMC-treated animals presented higher levels of TGF-β and IL-10 than untreated animals on day 70 [11]. These conflicting results regarding TGF-β expression might be attributed to its kinetics after silica instillation and to the time point of cell-based therapy. A previous study from another group has shown that TGF-β presented lower levels at the early stage and reached peak concentration in the chronic stage of a murine model of pulmonary tuberculosis [32]. Moreover, increased levels of TGF-β may be associated with a T regulatory response, because TGF-β and IL-10 secreted by regulatory T cells can suppress Th1 immune response, which leads to a preferential Th2 response in murine silicosis [33]. In the present study, BMMC-healthy and BMMC-sil therapies differently modulated TGF-β and IL-10 protein levels, which might be attributed to changes in regulatory T cell recruitment, since BMMC-healthy therapy led to an increased number of FoxP3^+^ T cells in lung tissue in the late stage of the disease [11].

The article "Therapeutic effects of bone marrow-derived mononuclear cells from healthy or silicotic donors on recipient silicosis mice" was published in 2017. Journal: Stem Cell Res Ther.

Pulmonary fibrosis occurs when collagen synthesis overwhelms degradation of ECM components [7], leading to tissue remodeling and impairment of lung function [34]. In the present study, we observed that silicotic animals presented increased TGF-β levels as well as collagen deposition in lung tissue. Administration of BMMC-healthy, but not BMMC-sil, reduced silica-induced lung fibrosis, possibly by reducing TGF-β levels. Moodley et al. [21] have previously observed that reduction in collagen synthesis after cell-based therapy is directly associated with reduction in TGF-β levels in a murine model of bleomycin-induced lung fibrosis, corroborating our results in experimental silicosis.

To better understand the effects of BMMCs on lung fibrosis in our model of silicosis, we evaluated mRNA expression of MMP-9 and type III and I procollagen, which are abundant in the early and late phases of lung remodeling. In the present study, the BMMC-sil-treated group presented reduced mRNA expression of type III and I procollagen, which could be associated with lower MMP-9 expression. A previous study analyzing the plasma levels of TNF-α and MMP-9 in patients with silicosis has suggested that both molecules have higher expression in the early course of silica exposure [35]. In addition, Ramos et al. [36] have reported that lung fibroblasts obtained from patients with idiopathic pulmonary fibrosis strongly express α1-(I) collagen and MMP-9, which demonstrates their importance in lung fibrosis progression [36]. Moreover, the effects of cell therapy on collagen deposition were previously correlated to reduced expression of MMP-2, MMP-9, and MMP-13 [20]. Therefore, our results suggest that BMMC therapy acts by systemic release of mediators that reduce the secretion of fibrotic factors and then prevent fibroblast activation and collagen deposition in lung parenchyma.

The article "Therapeutic effects of bone marrow-derived mononuclear cells from healthy or silicotic donors on recipient silicosis mice" was published in 2017. Journal: Stem Cell Res Ther.

In addition to the effects of TGF-β on silica-induced lung fibrosis, the increased apoptotic cell counts in lung parenchyma have been correlated to increased TGF-β levels [11, 27, 37]. Some studies that carried out BMMCs transplantation have demonstrated anti-apoptotic effects in different experimental models [38, 39], and a previous study from our group has shown that repeated administration of bone marrow-derived cells reduced mRNA expression of pro-caspase 3, as well as apoptotic cell counts in lung parenchyma and granulomas [40]. Here, we have observed that both BMMC-healthy and BMMC-sil reduced apoptotic cell counts in the lung parenchyma, but not in granulomas.

Our group has recently reported a phase I clinical trial of intrabronchial instillation of BMMCs in patients with silicosis, which to our knowledge is the first clinical study evaluating the safety of cell-based therapy in silicosis [41]. In that study, we observed that (1) there were no adverse effects during and after BMMC administration; (2) lung function, quality of life, and radiologic features remained stable throughout follow-up; and (3) an early increase in perfusion in the base of both lungs after BMMC administration. The experimental setting used in the present study mimics autologous BMMCs therapy. This allow us to understand the beneficial effects of cell-based therapy, since the murine model of silicosis reproduces the changes observed in patients with silicosis, using a short-term protocol.

## Conclusions

Administration of BMMCs obtained from both healthy and silicotic donors led to morpho-functional improvement in silicotic animals by differently modulating inflammatory and fibrogenic processes in the lungs. Our results indicate that BMMCs therapy acts by releasing mediators systemically, which mitigate the inflammatory and remodeling processes, ultimate leading to improvement in lung function. Although we did not observe differences in the profile of the BMMCs population from healthy and silicotic donors, administration of BMMC-healthy seems to have a greater effect by decreasing F4/80^+^ macrophage cell counts, IL-1β protein levels in lung tissue, and collagen content in experimental silicosis.

The article "Therapeutic effects of bone marrow-derived mononuclear cells from healthy or silicotic donors on recipient silicosis mice" was published in 2017. Journal: Stem Cell Res Ther.

## Abbreviations

BMMC: Bone marrow mononuclear cell
CT: Computed tomography
DMEM: Dulbecco’s modified Eagle’s medium
ECM: Extracellular matrix
GFP: Green fluorescent protein
HSC: Hematopoietic stem cell
IL-1β: Interleukin-1 beta
MMP: Matrix metalloproteinase
MSC: Mesenchymal stem cell
PCR: Polymerase chain reaction
SD: Standard deviation
TGF-β: Transforming growth factor beta
TNF-α: Tumor necrosis factor alpha.
